The article "Accelerated Aging Effects on Color Change, Translucency Parameter, and Surface Hardness of Resin Composites" was published in 2022. Journal: Biomed Res Int.

# Accelerated Aging Effects on Color Change, Translucency Parameter, and Surface Hardness of Resin Composites

**DOI:** 10.1155/2022/6468281

**Published:** 2022-08-02

**Authors:** Muhammet Fidan

**Affiliations:** Department of Restorative Dentistry, Faculty of Dentistry, Usak University, Usak, Turkey

## Abstract

**Background:**

The aging process can induce a change in the surface microstructure of materials, the chemical compositions of matrices, and the filler particles of resin composites. This study is aimed at evaluating the effects of accelerated artificial aging (AAA) on the color change, translucency parameter (TP), and surface hardness of resin composites.

**Methods:**

Five resin composite materials (Tetric N-Ceram, Filtek Z250, Charisma Smart, Herculite Classic, and Escom100) were evaluated. A spectrophotometer was used for color measurements (*L*∗, *a*∗, and *b*∗). TP and color changes (Δ*E*_00_) were calculated using the CIEDE2000 formula. The resin materials were subjected to aging for 300 hours. The hardness and TP values were measured before and after AAA. One- and two-way ANOVA and the Tukey test were used. The significance level was accepted as *p* < 0.05.

**Results:**

Escom100 had significantly higher Δ*E*_00_ values than the other resin composites, and Charisma Smart had significantly lower Δ*E*_00_ values than the other tested materials (*p* < 0.05). Before and after AAA, Charisma Smart had the lowest TP values, and Filtek Z250 exhibited the highest hardness values (*p* < 0.05). For TP and surface hardness, the effect size value of the composite material was found to be higher than that of AAA.

**Conclusions:**

After AAA, the investigated resin composites had Δ*E*_00_ values that were above clinically acceptable thresholds. After aging, the tested materials generally exhibited decreases in *L*∗ values and *a*∗ values, while increases in *b*∗ values were observed. The *Δ*TP values of the resin composites were similar. AAA significantly increased the surface hardness of the tested materials.

## 1. Introduction

Efforts in dental restorative material innovation have largely emphasized the emulation of the aesthetic and mechanical properties (including color and surface texture) of natural teeth as closely as possible [1]. Restorative materials mainly consist of inorganic and organic filler particles, as well as photoinitiators, accelerators, and pigments. However, these materials may deteriorate over time, consequently affecting the appearance and durability of resin composites. Color stability of resin materials is an important aesthetic feature of restorative materials [2]. Notably, significant discoloration is an important and common indication that dental restorations need to be replaced [3].

The article "Accelerated Aging Effects on Color Change, Translucency Parameter, and Surface Hardness of Resin Composites" was published in 2022. Journal: Biomed Res Int.

Translucency is an optical property that lies between opacity and transparency in terms of the amount of light that can pass through a material. Unlike transparent materials, translucent materials scatter light rays and prevent objects behind the material from being seen clearly [4]. The translucency parameter (TP) is used to assess the translucency of restorative materials. The translucency of resin composite materials is affected by their color, thickness, and material composition. In most translucency studies in the dental literature, translucency has been measured using the CIELAB color formula [5]. Some researchers have advocated the use of the CIEDE2000 color formula, which aims to correct and improve the perceived and calculated color differences determined by the CIELAB color formula [6, 7].

Surface hardness is a mechanical property that plays an important role in the durability of dental restorations [1]. However, filler volume and size, differences in matrix composition, and changes in polymerization technology can affect mechanical and physical properties [8]. Understanding the mechanical durability of restorative materials is important for the successful application of posterior restorations. The forces acting on dental restorations have direct effects on durability and can cause fractures in the restoration and/or underlying tooth. Oral cavity factors such as light, humidity, pH, temperature, pressure, and mechanical wear, as well as the interactions between these factors, can deteriorate and age dental restorations [9].

*In vitro* studies were performed to simulate clinical situations as closely as possible within the scope of clinical procedures [10]. Accelerated artificial aging (AAA) can be applied to materials as a proxy for long- or short-term deterioration that may lead to changes in these materials' mechanical and optical properties [3]. AAA is among the most widely used methods to simulate the aging process of resin composites in the oral environment over time [11]. AAA mimics environmental factors, such as lights, temperatures, and humidity. Ideally, the effects of AAA are equivalent to the effects of long-term use [12]. The aging method can cause changes in the microstructure of materials, the compositions of matrices, and the filler particles of resin composites [13]. Moreover, AAA can degrade resin matrices by promoting the degradation of resin composites and changing the structural distribution of the particles, negatively affecting the materials' mechanical properties [14]. AAA can alter optical and mechanical properties. An examination of the relevant literature has not shown the magnitude of the effects of AAA. This study was aimed at evaluating the effects of AAA on the color, TP, and hardness of composite materials. The null hypothesis is that AAA does not influence the color change, TP, and hardness of the investigated resin composites.

The article "Accelerated Aging Effects on Color Change, Translucency Parameter, and Surface Hardness of Resin Composites" was published in 2022. Journal: Biomed Res Int.

## 2. Materials and Methods

Shade A1 of five different resin composites (Tetric N-Ceram, Ivoclar Vivadent, Schaan, Liechtenstein; Filtek Z250, 3M-ESPE, St. Paul, MN, USA; Herculite Classic, KerrHawe, Bioggio, Switzerland; Escom100, Spident, Gojan-dong, Namdong-gu, Incheon, Korea; Charisma Smart, Heraeus Kulzer, Hanau, Germany) were used (Table 1). A Teflon mold (8 mm diameter-2 mm thickness) was used to create disc-shaped samples of the resin composite materials. Resin composites were polymerized with curing light (Woodpecker LED.E (P), Woodpeckers Med. Inst. Co., Guilin, China) at 1200 mW/cm^2^ for 40 seconds over Mylar strips. Twenty disc-shaped samples were created for each resin group. For standardization, a polishing system (OptiDisc, KerrHawe, Bioggio, Switzerland) was used for a single surface of the samples, and each was used for 10 seconds in dry conditions. All samples were stored at 37°C for 24 hours in distilled water (Nuve Incubator, EN 055, Ankara, Turkey).

The baseline color measurements were obtained with a spectrophotometer (Lovibond RT Series, Tintometer Group, Lovibond House, UK). Three color measurements were made from each sample, and these measurements were averaged for each sample. The color differences were calculated using the CIEDE2000 formula [15, 16]:

(1) $$\begin{array}{c} \Delta E_{00}={\left[{\left(\frac{\Delta L^{\prime }}{K_{L}S_{L}}\right)}^{2}+{\left(\frac{\Delta C^{\prime }}{K_{C}S_{C}}\right)}^{2}+{\left(\frac{\Delta H^{\prime }}{K_{H}S_{H}}\right)}^{2}+R_{T}\left(\frac{\Delta C^{\prime }}{K_{C}S_{C}}\right)\left(\frac{\Delta H^{\prime }}{K_{H}S_{H}}\right)\right]}^{1/2}, \end{array}$$

where Δ*L*′, Δ*C*′, and Δ*H*′ are the change in lightness, chroma, and hue, respectively, between the two specimens. The relationship between the variations of chroma and hue in the blue region is defined by the rotation function (*R*_*T*_). The weighting functions of lightness, chroma, and hue are denoted by *S*_*L*_, *S*_*C*_, and *S*_*H*_, respectively. *K*_*L*_, *K*_*C*_, and *K*_*H*_ are the parametric factors of set 1 in this study [6, 17].

For TP, the baseline color measurements were obtained with a spectrophotometer (Lovibond RT Series, Tintometer® Group, Lovibond House, UK). TP was calculated using the CIEDE2000 formula [5]:

(2) $$\begin{array}{c} {TP}_{00}={\left[{\left(\frac{{L_{B}}^{\prime }-{L_{W}}^{\prime }}{K_{L}S_{L}}\right)}^{2}+{\left(\frac{{C_{B}}^{\prime }-{C_{W}}^{\prime }}{K_{C}S_{C}}\right)}^{2}+{\left(\frac{{H_{B}}^{\prime }-{H_{W}}^{\prime }}{K_{H}S_{H}}\right)}^{2}+R_{T}\left(\frac{{C_{B}}^{\prime }-{C_{W}}^{\prime }}{K_{C}S_{C}}\right)\left(\frac{{H_{B}}^{\prime }-{H_{W}}^{\prime }}{K_{H}S_{H}}\right)\right]}^{1/2}. \end{array}$$

Subscripts “*B*” and “*W*” (specified in the formula) correspond to black and white backgrounds, respectively. (*L*_*B*_′ − *L*_*W*_′), (*C*_*B*_′ − *C*_*W*_′), and (*H*_*B*_′ − *H*_*W*_′) denote the changes in lightness, chroma, and hue on black and white backgrounds, respectively. The relationship between the variations of chroma and hue in the blue region is defined by the rotation function (RT). The weighting functions of lightness, chroma, and hue are denoted by *S*_*L*_, *S*_*C*_, and *S*_*H*_, respectively. *K*_*L*_, *K*_*C*_, and *K*_*H*_ are the parametric factors of set 1 in this study [5, 17].

The article "Accelerated Aging Effects on Color Change, Translucency Parameter, and Surface Hardness of Resin Composites" was published in 2022. Journal: Biomed Res Int.

The baseline surface hardness was measured using a surface hardness device (LHV-1D, Bursam NDT, Bursa, Turkey). A 300 g load with a 15 s dwell period was used on the surface for three measurements, and the mean value was calculated for each material. After initial measurements, the resin composites were subjected for 300 h at 150 kJ/m^2^ in an aging chamber (Atlas ci 4000; Atlas Electronic Devices Co., Mount Prospect, USA) [18]. The aging procedure was performed as described in the previous study as follows [19]: 60 minutes in the dark with back water spray, 40 minutes under illumination, 20 minutes under illumination water spray, and 60 minutes under illumination. The temperature of the back panel was maintained at 38 ± 2°C in the dark and 70 ± 3°C under illumination. The dry-bulb temperature was 38 ± 2°C in the dark and 47 ± 3°C under illumination. Relative humidity was maintained at 95 ± 5% in the dark and 50 ± 5% under illumination [17]. After AAA, the procedures for measuring color change, TP, and hardness were repeated. SPSS Statistics for Windows, Version 22.0 (IBM Corp, Armonk, NY, USA) was used for the statistical analyses of data. The data were checked for normal distribution (Kolmogorov-Smirnov test-skewness kurtosis) and homogeneity (Levene test). Tukey's test was used for multiple comparisons. The Δ*L*, Δ*a*, Δ*b*, Δ*E*_00__,_ and *Δ*TP data were analyzed using a one-way analysis of variance (one-way ANOVA). A two-way ANOVA was used to determine the surface hardness and TP for main effects (composite, AAA) and the interaction between the factors (AAA∗composite). The Bonferroni correction was used to compare the main effects. Partial eta squared (*η*^2^) was used to rank the effect of independent variables on dependent variables when a two-way ANOVA was used. The significance level was accepted as *p* < 0.05.

The article "Accelerated Aging Effects on Color Change, Translucency Parameter, and Surface Hardness of Resin Composites" was published in 2022. Journal: Biomed Res Int.

## 3. Results

The tested composites generally exhibited a decrease in *L*∗ values and *a*∗ values and an increase in *b*∗ values after AAA (Table 2). Table 2 shows the Δ*E*_00_ values. Escom100 had significantly higher Δ*E*_00_ values than all other tested composites (*p* < 0.001). Δ*E*_00_ values of Charisma Smart were significantly lower than all other materials (*p* < 0.001).

Main effects and interactions (AAA, composite, and AAA × composite) on TP are shown in Table 3. No significant difference was found between AAA × composite interaction (*p* = 0.236). The main effect of AAA and composite on the TP values was significant (*p* values < 0.001 and <0.001, respectively) (Table 3). The TP value differences are shown in Table 4. Charisma Smart had the lowest TP values between tested materials (*p* < 0.001). Escom100 and Charisma Smart had the highest TP values between the tested materials. The TP of Filtek Z250 and Tetric N-Ceram were similar values (Table 4). The effect size of the AAA (*η*^2^ = 0.355) and the composite (*η*^2^ = 0.473) was found (Table 3).

The AAA, composite, and AAA × composite on the surface hardness values were found to be significant (*p* values < 0.001, < 0.001, and < 0.001, respectively) (Table 5). AAA significantly increased the hardness values of the investigated resin composites (*p* < 0.001). The surface hardness differences are shown in Table 6. Before and after AAA, among all resin composites, Filtek Z250 exhibited the highest hardness values (*p* < 0.001). The effect size for the AAA (*η*^2^ = 0.949) and the composite (*η*^2^ = 0.982) was found (Table 5).

## 4. Discussion

AAA significantly influenced the color change, TP, and surface hardness of resin composites. Therefore, the null hypothesis was rejected. In clinical contexts, dental materials are exposed to many factors, such as temperature, humidity, and mechanical stress, and must remain stable against these factors. *In vitro* testing is an inexpensive technique that can be used to predict material reliability [10]. Accelerated aging causes changes (deterioration) in the mechanical and optical properties of restorative materials [3]. AAA includes factors such as light, temperature, and humidity that cause amine oxidation [20]. The double bonds in aromatic amines can cause the yellowing of resins because these structures can absorb light from the device; higher energy can be generated, and these molecules react with the oxygen in the aromatic groups to form structures with higher energy [21]. During polymerization, temperature or light can cause initiators and tertiary aromatic amines to form products that cause resins to turn red or yellow [3]. This is consistent with previous studies wherein materials tested after accelerated aging generally exhibited decreases in *L*∗ and *a*∗ values and increases in *b*∗ values [10, 22]. In this study, the tested materials exhibited decreases in *L*∗ coordinate values, decreases in *a*∗ coordinate values, and increases in *b*∗ coordinate values (except for Herculite Classic).

The article "Accelerated Aging Effects on Color Change, Translucency Parameter, and Surface Hardness of Resin Composites" was published in 2022. Journal: Biomed Res Int.

In this study, the acceptable perceptibility and acceptability thresholds were 0.81 and 1.77, respectively [16]. Color change Δ*E*_00_ values were all between 2.1 and 5.9, and the investigated resin composites were associated with clinically unacceptable color changes after AAA. Escom100 showed the highest color change after AAA. Escom100 contains urethane dimethacrylate, which has been shown to be prone to yellowing after AAA [3]. The increase in the *b* value of Escom100 was significantly higher than that for the other composites. This color change may have been more drastic because of the interaction of AAA with the monomer structure in this material. The color change was observed to be visual yellowing, which is noted as the overall darkening of the resin materials during ultraviolet light illumination in laboratory experiments [17, 23]. Unlike other composites, Herculite Classic showed a tendency toward the color blue. It is thought that this may be due to pigments in the material affected by AAA. Celik et al. [24] stated that submicron hybrid resin composite materials showed less color change than nanohybrid resin composite materials. In this study, the submicron hybrid composite (Charisma Smart) had significantly lower Δ*E*_00_ values than the nanohybrid and microhybrid resins. The better color stability of the material in the submicron content can be attributed to the organic filler sizes [24]. This is expected to contribute to a reduction in color degradation. However, a smaller filler size does not necessarily equate to less staining [17, 25]. The color stability of resin materials is related to the matrix and filler composition and content, macroscopic phenomena, pigmentation, purity of the oligomers and monomers, the concentration/type of activators, initiators, inhibitors, and the oxidation of unreacted carbon–carbon double bonds [24]. The degradation of residual amines and oxidation of residual unreacted carbon–carbon double bonds results in yellowing of resin composites [25], as the increased yellowing of nanocontaining composites is presumed to be due to a lower degree of conversion or aging process.

The TP of a material is defined by its difference in color on a white and black background [3]. The translucency of a material is related to the extent or abundance of absorption, light scattering, organic matrix, and filler particles [17, 26]. AAA decreased the TP values of the resin composite materials used in this study. However, there were no significant differences in *Δ*TP values among the resin composite materials. This finding is consistent with that of a previous study that found that AAA does not affect *Δ*TP values [3]. The translucency of restorative materials depends on absorption and scattering, which occurs due to refractive index mismatches in the organic matrix and filler particles vs. the size and dispersion of inorganic fillers [27]. Azzopardi et al. [28] found that resin matrix and filler particles could affect the translucency of experimental resin composites. Other studies have shown that nanohybrid composite resins have high translucency due to particle sizes smaller than the wavelength of light, resulting in minimal scattering of photons [29, 30]. In this study, Escom100 had higher TP values than the other investigated materials, probably due to differences in light scattering resulting from Escom100's nanosized filler particles. Charisma Smart had the lowest TP values in our study. This can be attributed to the composition of this submicron material. The translucency, opacity, and light transmission properties of resin composites are influenced by resin matrix composition, pigments, and other added substances, which result in light reflection at different wavelengths [31, 32]. Howard et al. [33] found that the differences in refractive indices between fillers and matrices decrease with an increase in the carbon–carbon double bond conversion degree of monomers; thus, resin scatters more light and is more translucent. Material content differences can be attributed to variations in TP values. Translucency values are affected by many factors, such as the content of the applied resin matrix [5], resin matrix content [28], distribution of fillers, and types of polymerization initiators and inhibitors [34]. In resin composite materials, light absorption is enabled by the organic matrix, while diffusion occurs because of the size and distribution of inorganic fillers and the difference between the refractive index of the organic matrix and inorganic fillers [35]. In this context, the differences in material contents in our study reflect differences in TP values. AAA influences the filler particles related to the reflection and transmission of light by changing the perceptions of translucency [3, 17]. This may explain the decrease in TP values after AAA. The effect size of the composite was higher than that of the AAA effect [17]. This finding indicates that the content of composites has a higher effect size on TP values than AAA.

The article "Accelerated Aging Effects on Color Change, Translucency Parameter, and Surface Hardness of Resin Composites" was published in 2022. Journal: Biomed Res Int.

Hardness is an important mechanical property [36], as surface hardness affects wear [37] and can increase surface roughness in soft materials. This can cause color changes, secondary caries, plaque formation, and gingival inflammation [36]. The microhardness of a material can be influenced by the type, shape, and size of the fillers, as well as the chemical properties [38]. In our study, zirconia particles may have affected the increase in the hardness values of Filtek Z250. A previous study [14] found that among different resin composites, the composite material (Z250-microhybrid) with silica and zirconia content was the hardest. Another study showed that the mechanical properties of the prepolymerized structure contained in Charisma Smart might be weak [36]. Tetric N-Ceram had the lowest hardness values before and after AAA in our study. This may be due to its prepolymerized structure [39]. The hardness of resin composites depends on several factors, such as the content of the resin matrix and the types and shape of the particles. Moreover, the hardness of resin composite is directly related to filler particles [40]. A previous study reported that there was a significant decrease in the microhardness values of resin composite materials after AAA [41]. In contrast, Rattacaso et al. [42] demonstrated an increase (after AAA) in the Knoop microhardness values of the resin composite materials evaluated in their study. Another study found that AAA did not affect the hardness values of resin composites, but there were significant differences in hardness values between materials [14]. In our study, the hardness values of the investigated resin composites significantly increased after AAA, as postpolymerization was caused by an increase in temperature and water condensation [42]. The factors applied in accelerated aging may increase the hardness of the materials. Characterization analyses of the materials should be performed to improve the understanding of mechanical behavior. The composite effect size was higher than the AAA effect. This finding indicates that the composite contents have a higher effect size on surface hardness than AAA.

An attempt was made to simulate the oral environment within the methodological limitations of this study. AAA is designed to simulate sunlight and accelerated degradation by UV stress, but since the mouth is closed most of the time rather than open, UV stress is rarely applied to composite resins and constitutes a limitation of this study. Saliva, temperature changes, and pH levels in the mouth, along with patient habits and brushing, can also affect the optical and mechanical properties of resin composite materials. Based on our findings, we can conclude that the optical and mechanical properties of the investigated materials are affected by AAA. Further studies should be conducted to examine the effects of different degrees of aging on the optical and mechanical properties of resin composites.

The article "Accelerated Aging Effects on Color Change, Translucency Parameter, and Surface Hardness of Resin Composites" was published in 2022. Journal: Biomed Res Int.

## 5. Conclusion

After AAA, the investigated resin composites had Δ*E*_00_ values that were above clinically acceptable thresholds. The submicron composite (Charisma Smart) exhibited better color stability after AAA. The tested materials exhibited decreased *L*∗ and *a*∗ values, along with increased *b*∗ values (except for Herculite Classic). The *Δ*TP values of the resin composites were similar. AAA significantly increased the hardness values of resin composites. The composite had a higher effect size on the surface hardness and TP than AAA. Clinicians should thus be cognizant of the content of resin composites.

## Figures and Tables

**Table 1:** List of materials used in present study.

Resin composites	Manufacturer	Type	Composition	Volume	Lot no.
Filtek Z250	3M Espe, St. Paul, MN, USA	Microhybrid	BisGMA, UDMA, Bis-EMA, zirkonium/silica, 0,01-3,5 *μ*m	60%	NA41529
Tetric N-Ceram	Ivoclar Vivadent, Schaan, Liechtenstein	Nanohybrid	Bis-GMA, UDMA, BisEMA, barium glass, prepolymer, ytterbium trifluoride, mixed oxide, copolymers, 40-3000 nm	77%	W14342
Charisma Smart	Heraeus Kulzer, Hanau, Germany	Submicron-hybrid	Bis-GMA, barium-aluminum-fluoride glass, silicon dioxide, 0.005-10 *μ*m	59%	K010516
Herculite Classic	KerrHawe, Bioggio, Switzerland	Microhybrid	Bis-GMA, TEGDMA, camphorquinone, amine, iron oxide pigments, aluminum borosilicate glass, colloidal silica	59%	6933034
Escom100	Spident, Gojan-dong, Namdong-gu, Incheon, Korea	Nanohybrid	UDMA, barium glass	75-80%	E1A17031

Bis-GMA: bisphenol A glycol dimethacrylate; Bis-EMA: bisphenol A ethoxylated dimethacrylate; TEGDMA: triethylene glycol dimethacrylate; UDMA: urethane dimethacrylate.

**Table 2:** Means and standard deviations for differences in Δ*L*, Δ*a*, Δ*b*, and Δ*E*_00_ (Δ*L*, Δ*a*, and Δ*b*; baseline minus after accelerated aging).

Resin composites	Δ*L*	Δ*a*	Δ*b*	Δ*E*_00_
Filtek Z250	-3.98 (1.41)^A^	-0.08 (0.63^A^	4.11 (3.65)^A^	3.96 (1.26)^A^
Tetric N-Ceram	-3.11 (1.09)^AB^	-0.85 (0.30^B^	3.77 (1.38)^A^	3.52 (0.81)^A^
Charisma Smart	-2.70 (1.26)^B^	-0.21 (0.24^A^	0.48 (1.20)^B^	2.11 (0.77)^B^
Herculite Classic	-2.69 (1.60)^B^	-1.65 (0.20)^C^	-3.87 (1.28)^C^	4.17 (0.62)^A^
Escom100	-5.21 (1.02)^C^	−1.26 ± (0.45)^D^	7.47 (0.97)^D^	5.90 (0.66)^C^

Different capital letters represent statistically significant differences in each column (*p* < 0.05).

The article "Accelerated Aging Effects on Color Change, Translucency Parameter, and Surface Hardness of Resin Composites" was published in 2022. Journal: Biomed Res Int.

**Table 3:** Two-way ANOVA results main effects and interaction for TP.

Source	Type III	df	Mean square	*F*	*p*	Partial eta squared
AAA	67.611	1	67.611	104.665	<0.001	0.355
Composite	110.321	4	27.580	42.696	<0.001	0.473
Composite ∗ AAA	3.611	4	0.903	1.398	0.236	0.029

a.R squared = .597 (adjusted R squared = .578).

**Table 4:** Means and standard deviations for TP and *Δ*TP (baseline minus after accelerated aging) of the tested materials.

Resin composites	Before AAA	After AAA	Total (composite)	*Δ*TP∗
Filtek Z250	7.70 (0.70)	7.03 (0.95)	7.37 (0.89)^a^	-1.18 (0.66)^a^
Tetric N-Ceram	8.24 (0.73)	6.77 (0.82)	7.51 (1.07)^a^	-1.46 (0.99)^a^
Charisma Smart	6.86 (0.90)	5.59 (0.75)	6.23 (1.04)^b^	-1.46 (0.95)^a^
Herculite Classic	8.74 (0.80)	7.47 (1.03)	8.11 (1.08)^c^	-1.26 (0.96)^a^
Escom100	8.94 (0.43)	7.79 (0.82)	8.37 (0.87)^c^	-1.15 (0.76)^a^
Total (AAA)	8.09 (1.03)^A^	6.93 (1.15)^B^	7.52 (1.24)	

Different capital letters represent statistically significant differences in each row (*p* < 0.05) (main effect; AAA). Different lower letters represent statistically significant differences in each column (*p* < 0.05) (main effect; composite). There is no difference between the interaction factors (*p* > 0.05) (AAA∗composite). ∗*Δ*TP: there is no difference between the composites.

**Table 5:** Two-way ANOVA results for surface hardness main effects and interaction.

Source	Type III	df	Mean square	*F*	*p*	Partial eta squared
AAA	14392.43	1	14392.427	3522.51	<0.001	0.949
Composite	42110.63	4	10527.657	2576.61	<0.001	0.982
Composite ∗ AAA	1363.54	4	340.884	83.43	<0.001	0.637

a.R squared = .987 (adjusted R squared = .986).

**Table 6:** Means and standard deviations for surface hardness of the tested materials.

Resin composites	Before AAA	After AAA	Total (composite)
Filtek Z250	89.25 (2.09)^A^	104.06 (4.03)^A^	96.65 (8.14)^a^
Tetric N-Ceram	47.60 (1.84)^B^	66.13 (1.55)^B^	56.87 (9.53)^b^
Charisma Smart	51.96 (2.15)^C^	67.36 (1.58)^B^	59.66 (8.01)^c^
Herculite Classic	59.76 (0.99)^D^	69.92 (1.42)^C^	64.84 (5.28)^d^
Escom100	49.70 (1.50)^E^	75.64 (1.40)^D^	62.67 (9.20)^e^
Total (AAA)	59.65 (15.53)^a^	76.62 (14.34)^b^	68.14 (17.16)

?Different lower letters represent statistically significant differences from before and after total hardness values in each row *p* < 0.05 (main effect; AAA). Different lower letters represent statistically significant differences from total composites hardness values in each column *p* < 0.05 (main effect; composite). ^A-E^There is no difference between the same capital letter (interaction; AAA∗composite).

## Data Availability

The datasets used and analyzed during the current study are available from the corresponding author upon reasonable request.
